# TAP Test Image Dynamic Tracking Study after Thyroid Cancer Surgery and after Radiotherapy and Chemotherapy

This article has been retracted.

**DOI:** 10.1155/2021/8072126

**Published:** 2021-04-16

**Authors:** Changliang Wang, Yongxue Gu, Xiaojuan Men, Peng Sun, Meili Chen

**Affiliations:** ^1^Department of Galactophore Surgery, Weifang People's Hospital, Shandong 261041, China; ^2^Weifang Medical University, Shandong 261041, China; ^3^Weifang Brain Hospital Emergency Department, Shandong 261041, China

## Abstract

Thyroid cancer is a relatively common endocrine gland malignant tumor; if improper treatment, there will be a high risk of recurrence or metastasis, and abnormal sugar chain glycoprotein (TAP) has a close relationship with the development of the disease; therefore, the purpose of this article is to discuss abnormal sugar chain glycoprotein (TAP) as thyroid cancer curative effect evaluation and radiation and chemotherapy after surgery clinical significance. In this paper, 95 patients with thyroid cancer diagnosed in a hospital were selected as the study objects and treated as the observation group. The clinical and follow-up data of the observation group were retrospectively analyzed. Meanwhile, 55 healthy patients were randomly selected as the control group. TAP, squamous cell carcinoma antigen (SCC) level, and carcinoembryonic antigen (CEA) level were detected in peripheral blood of 95 patients with thyroid cancer before and after treatment. The short-term efficacy was evaluated by chest CT examination, and the changes of the three markers before and after treatment and the correlation with the short-term efficacy of the patients were compared. According to the results of testing, the TAP positive expression in patients before radiotherapy can better predict the recent curative effect has certain clinical value; before radiotherapy TAP positive expression rate was significantly higher than that of healthy people, TAP positive expression quantity decreased obviously after radiation treatment, and patients with a recent radiotherapy curative effect is good or bad and negatively correlated with the degree of TAP protein positive expression; TAP high protein in patients with recent poor radiation effects, prompt the factor can be predicted in the near future curative effect of the molecular markers, and can TAP level for clinicians provide certain reference for targeted therapy.

## 1. Introduction

The incidence of thyroid cancer is increasing year by year, and the age of onset is getting younger [1, 2], which is a relatively common malignant tumor [3]. Early thyroid cancer with no obvious symptoms or signs was mostly found in the form of thyroid nodules in physical examination [4]. Current clinical though an ultrasound examination and puncture pumping fine needle biopsy detection methods, such as [5, 6], but some patients still cannot determine the nature of the lesion and the need to closely follow up even choose surgical resection in order to avoid delay in diagnosis or treatment, which has increased the psychological burden of patients and physical trauma, so looking for tumor markers to assist in the diagnosis of benign and malignant thyroid nodule has important significance. Abnormal glucose-chain glycoprotein (TAP) is an abnormal complex that occurs in the malignant transformation stage of cells and is expressed after mutations of oncogenes and tumor suppressor genes. When cancer cells proliferate abnormally, TAP is released into the blood and is mostly in peripheral blood [7]. TAP test is a one-time combination detection of up to dozens of abnormal sugar chain proteins related to tumors, with high sensitivity and accuracy. TAP test has been widely used in the screening and diagnosis of malignant tumors of the digestive system, breast, and gynecology but, rarely, reported in the diagnosis of thyroid cancer.

One-third of malignant tumors can be prevented, one-third can be cured if diagnosed early, and one-third can alleviate and prolong life [8]. The prevention and treatment of tumor mainly focuses on prevention and the combination of prevention and treatment [9]. In patients with early-stage tumors, the number of cancer cells is still at a reversible stage in the development of the tumor, the blood vessels that feed the tumor have not yet developed, and the tumor tissue is still fragile. Malignant tumors are the product of complex factors and gene mutations [10]. For a normal cell to accumulate these “three” changes, it generally takes a long time (many years of undetectable initial period). This provides valuable time and opportunity for early detection and effective blocking of tumors. There are three clinical methods for early detection and diagnosis: physical methods (X-ray, b-ultrasound, CT, MRI, PET-CT, etc.), biochemical tests (such as blood lipid and glucose), and histopathological examination [11–13]. Currently, the most accurate instruments can only detect tumors in diameter of >0.5 cm. When the tumor mass from asymptomatic and gradually grow to be found by imaging, endoscopy and other examination is usually the clinical stage of the tumor, which has lost the optimal treatment period. That is to say, although these methods can assist the diagnosis and observation of tumors from different perspectives and to different degrees, they cannot fundamentally solve the problem of early detection and diagnosis of tumors. Domestic and foreign studies have shown that there is a close relationship between tumor marker TM and tumor [14, 15]. However, the sensitivity, specificity, and accuracy of a single TM test for tumor-assisted diagnosis or early diagnosis are poor, while TAP provides a new method for tumor diagnosis.

Scholars Li et al. assessed the level of the expression of CK20 and treatment effect and prognosis of postoperative colorectal cancer of correlation, the experiment to the postoperative follow-up of 62 patients with colorectal cancer, tumor tissue, and the abdominal cavity drainage liquid samples and blood sampling; in the fluid of the tumor specimens and abdominal cavity drainage, early cancer patients CK20 level lower than that of patients with advanced cancer, serum CK20 negative 3-year survival rate of patients was obviously higher than that of CK20 seropositive patients [16]. Scholars Wu and Huang discussed TAP and other serological biomarkers such as carcinoembryonic antigen (CEA), antigen 125 (CA125) sugar, and sugar antigen 19-9 (CA19-9) relationship, and its clinical application in patients with colorectal cancer (CRC) results showed that the TAP detection in CRC patients with high sensitivity and specificity of clinical monitoring in the process of CRC patients with chemotherapy can be used as a new independent index [17]. Scholars Li et al. combined TAP with hs-CRP level test to diagnose endometrial cancer in patients with endometrial thickness less than 8 mm. Their results showed that for suspected endometrial cancer patients with endometrial thickness less than 8 mm, the combined TAP and hs-CRP test could be used as a screening tool, providing new ideas for clinical diagnosis and treatment [18]. Scholar Fan studied the value of tumor markers C12 system in gastric cancer, using univariate and multivariate evaluation of tumor markers clinicopathologic correlation; using chi-square test to select key tumor markers in the diagnosis of gastric cancer is the most favorable combination; the result shows that the tumor marker biochip system has an important diagnostic value for gastric cancer, and CA19-9, CA242, CEA, and CA125 are four key indexes for tumor diagnosis [19]. Scholars Mo discusses the three tumor markers combined test value to the diagnosis of gastric cancer; the results showed that the levels of tumor markers gastric cancer group were obviously higher than that of control group; gastric cancer tumor markers combined detection sensitivity and accuracy were higher than pure detection, and CEA, CA199, and CA724 single detection has certain significance to the diagnosis of gastric cancer; the joint detection can improve the sensitivity and accuracy of diagnosis of gastric cancer [20]. Scholars Liu et al. studied the role of tumor markers in the differential diagnosis of benign and malignant ascites; the result shows that under the booking cutoff value of tumor markers, the diagnosis of ascites tumor markers' effect is better than that of the serum tumor markers; combined use of tumor markers and cytology can increase the diagnostic rate of the latter is 37%; in malignant ascites cytology negative, tumor markers are helpful to differentiate malignant ascites and benign ascites; ascites tumor markers are used in combination with sensitivity of 86%, specificity of 97%, which means that the detection of tumor markers may be useful auxiliary cytology [21]. Scholars Zhu et al. discussed in this paper the four kinds of tumor markers in serum and ascites and ascites/serum ratio value in the differential diagnosis of benign and malignant ascites, the experiment selected as the research object, and 76 patients divided into malignant ascites group (45 cases) and benign ascites group (31 cases); the experimental results show that compared with the single index, the joint detection in the serum and ascites tumor markers can significantly increase the sensitivity and specificity of diagnosis [22]. Scholars Trapé et al. studied the ascites tumor antigen 125 (CA125) and cytokeratin 19 soluble pieces (CYFRA21-1) and the tumor markers in the accuracy of the diagnosis of malignant ascites and analyzed 143 cases of patients with undiagnosed liver muscle inflammation CA125 and CYFRA21-1; the use of CA125 the sensitivity of the differential diagnosis of malignant ascites was 39.7% and specificity of 98.8%; the sensitivity of the differential diagnosis CYFRA21-1 was 50.0% and specificity of 97.6%, a combination of CA125 and CYFRA21-1. The sensitivity and specificity of these two tumor markers were 65.5% and 96.5%, respectively. In cytological negative patients, the sensitivity and specificity of these two tumor markers were 50% and 96.5%, respectively. The conclusion that the determination of tumor markers in treating ascites has a certain reference value for the diagnosis of ascites patients [23]. Scholars Cao and others studied the serum ALDH1A1 in nonsmall cell lung cancer diagnosis and prognosis of the potential clinical value in the experiment collected 100 patients with nonsmall cell lung cancer tumor resection before 60, 60 patients with benign lung disease and serum samples of healthy volunteers and using sandwich ELISA method were retrospectively analyzed, their results show that the levels of serum ALDH1A1 associated with the occurrence and progress of nonsmall cell lung cancer, and serum ALDH1A1 detection is helpful to the diagnosis and prognosis of nonsmall cell lung cancer. Combined application of carcinoembryonic antigen and ALDH1A1 can significantly improve the diagnostic rate of nonsmall cell lung cancer [24]. Xiao and other scholars studied the lung tissue and tumor markers in serum HE4 expression levels and its role in the differential diagnosis of lung cancer, the experiment tested the 214 cases of lung cancer patients and 76 cases of healthy human lung adenocarcinoma, lung squamous carcinoma, and adjacent tissues in the expression of HE4, and results show that the HE4 as a biomarker of lung cancer, for the early diagnosis of lung cancer, can provide important reference [25].

Thyroid cancer is a relatively common endocrine gland malignant tumor; if improper treatment, there will be a high risk of recurrence or metastasis, and abnormal sugar chain glycoprotein (TAP) has a close relationship with the development of the disease; therefore, the purpose of this article is to discuss abnormal sugar chain glycoprotein (TAP) as thyroid cancer curative effect evaluation and radiation and chemotherapy after surgery clinical significance. In this paper, 95 patients with thyroid cancer diagnosed in a hospital were selected as the study objects and treated as the observation group. The clinical and follow-up data of the observation group were retrospectively analyzed. Meanwhile, 55 healthy patients were randomly selected as the control group. TAP, squamous cell carcinoma antigen (SCC) level, and carcinoembryonic antigen (CEA) level were detected in peripheral blood of 95 patients with thyroid cancer before and after treatment. The short-term efficacy was evaluated by chest CT examination, and the changes of the three markers before and after treatment and the correlation with the short-term efficacy of the patients were compared. According to the results of testing, the TAP positive expression in patients before radiotherapy can better predict the recent curative effect has certain clinical value; before radiotherapy TAP positive expression rate was significantly higher than that of healthy people, TAP positive expression quantity decreased obviously after radiation treatment, and patients with a recent radiotherapy curative effect is good or bad and negatively correlated with the degree of TAP protein positive expression; TAP high protein in patients with recent poor radiation effects, prompt the factor can be predicted in the near future curative effect of the molecular markers, and can TAP level for clinicians provide certain reference for targeted therapy.

## 2. Thyroid Cancer and TAP Test

### 2.1. Diagnosis of Thyroid Cancer

It is well known that the possibility of thyroid cancer should be considered when the following clinical signs occur: rapid growth of thyroid nodules, hard texture, adhesion and fixation with surrounding tissues and organs, or regional lymph node enlargement. Especially solitary nodules occurring in childhood or male adults; thyroid nodules in patients with a history of head, neck, or chest radiotherapy; and thyroid nodules in patients with Grave's disease were characterized by low functional nodules on radionuclide scan and substantial masses on ultrasonography. Fine needle aspiration cytology (FNAC) should be performed in the above patients. In addition, the possibility of thyroid cancer should be suspected even if the following signs are clinically present.

#### 2.1.1. Cystic Masses

It is generally believed that thyroid tumor cystic or solid is helpful to benign and malignant diagnosis, even some people think that cystic masses malignant possibility is not big, in the treatment that often uses the simple cyst excision nor postoperative pathologic examination, leading to postoperative thyroid cancer relapses, is common: thyroid cancer actually can present a substantial, cystic, or mixed, and a report into the lumen of the mastoid shaped gland thyroid carcinoma tissues form can reach 45%~60% adenocarcinoma (sac). Malignant lesions accounted for 32% of the 60 cystic thyroid masses reported by Resent. Therefore, a cystic thyroid mass cannot exclude malignant lesions.

#### 2.1.2. Multiple Mass

Although thyroid cancer is dominated by a single nodule, the incidence of unilateral multicentric adenocarcinoma is reported to be 13%, and bilateral multicentric carcinoma is reported to be 6.0%-8.8%. Thyroid cancer, especially after radiotherapy, is often multicentric.

#### 2.1.3. Benign Thyroid Disease Coexists with Thyroid Cancer

In addition to thyroid adenoma and nodular goiter can be cancerous, thyroid can also coexist with some benign lesions. It was reported that 0.76%~8.7% of hyperthyroidism was associated with thyroid cancer, with a greater likelihood of toxic nodular goiter and high functional adenoma stage associated with thyroid cancer. The incidence of Hashimoto's disease with thyroid cancer is 5%~17%. There have also been reports of the coexistence of thyroid tumor and thyroid cancer.

Since it is very difficult to diagnose thyroid cancer before surgery, in cases requiring surgical treatment, no matter whether the diagnosis result is benign or malignant before surgery, patients with conditions should have a quick biopsy during routine surgery to determine the nature of pathology and guide the surgical method. The quality of frozen sections and the difference of thyroid cancer tissues may lead to false-negative results. Therefore, in addition to intraoperative frozen sections and rapid disease examination, routine paraffin sections should also be performed postoperatively to prevent missed diagnosis.

In addition, attention should be paid to thyroid microcarcinoma or occult carcinoma. Patients often seek treatment for swollen lymph nodes in the neck, but there are no clinical symptoms at this time. Therefore, patients with metastatic adenocarcinoma in the neck lymph nodes should carefully examine the thyroid gland.

### 2.2. Treatment of Thyroid Cancer

#### 2.2.1. Treatment Principles of Thyroid Cancer

The clinical manifestations, treatment methods, and therapeutic effects of different thyroid cancers are not completely the same. At present, it is generally accepted that the treatment plan should be determined according to the extent of thyroid primary lesion expansion, pathological type, and patient age, so as to achieve both radical treatment of the lesion and quality of life. The operation should include the primary lesion and the metastatic lesion in the neck. Although the choice of operation for thyroid cancer is still controversial, the current consensus is as follows.

#### 2.2.2. Selection of Primary Cancer Foci

Medullary carcinoma: total thyroidectomy and central lymph node dissection; undifferentiated cancer: preoperative diagnosed people generally do not advocate surgical treatment, only when the trachea is invaded, breathing difficulties, only consider surgery to remove the obstruction. If the postoperative pathological report is an undifferentiated tumor, radiotherapy should be added.

#### 2.2.3. The Choice of Surgical Method for Cervical Lymph Node Metastasis

At present, the vast majority of scholars advocate neck cleansing, generally do not advocate the use of preventive neck cleansing, such as bilateral metastasis, then phased neck cleansing.

#### 2.2.4. The Pathological Report after Thyroid Nodule Resection Was the Management of Thyroid Cancer

For patients who have undergone total lateral lobe resection, thyroxine inhibition therapy can be used under close observation. If subtotal resection of the affected lobe or local resection of the mass is performed, another operation should be performed immediately with the same surgical method as before. Because in the latter case, the residual gland has a high residual cancer rate.

#### 2.2.5. Radiotherapy after Surgery

Undifferentiated thyroid cancer is highly sensitive to external radiation therapy. Among the 305 cases of thyroid cancer reported in XiangYa hospital, 25 cases were undifferentiated. Among them, 7 underwent palliative surgery and received external radiation at 10-20 d after surgery. During follow-up, 5 patients survived for 18 to 24 months. Two cases survived for more than 2 years. In addition, 150 cases of well-differentiated thyroid cancer were treated with radiotherapy after surgery, and the 5, 10, and 15 survival rates were 76.19%, 56.25%, and 66.67%, respectively. Therefore, if there is no contraband, radiotherapy should be used after thyroid cancer, but myeloid cancer is not sensitive to radiotherapy.

### 2.3. TAP Detection

Glycoprotein (glycoprotein) is composed of two parts, protein and glycan connected by a covalent bond. Human cells can synthesize a certain type and amount of glycoprotein. Glycosylation of proteins is the most common modification after protein translation. Studies have shown that 1% of human genome involved in glycosylation and modification of sugar chains and about 70% of human proteins contain more than one sugar chain. Glycoprotein sugar chains are associated with a variety of biological processes, such as transport and processing of new peptide chains, interference with glycoprotein biological half-life, and influence on glycoprotein bioactivity and molecular recognition.

Oncogene and tumor suppressor gene mutations occur in human body. Malignant carcinogenesis is widespread abnormal glycosylation of membrane glycoproteins in the process of changes in cellular glycosyltransferase and colloidal enzyme activities. Modified proteins with abnormal changes in sugar chain structure are mainly represented by the new synthesis of sugar chains, and the hidden exposure of sugar chains is incomplete. After sugar chain synthesis, a variety of abnormal sugar chain glycoproteins are produced. When malignant cells approach a certain number, TAP produced by them is released into the blood and can be detected in peripheral blood.

At present, it is difficult to detect abnormal glycoprotein sugar chain directly. CLU is a group of sugar-binding proteins that can specifically recognize and bind to specific glycosyl sequences in a specific structural monosaccharide or oligosaccharide. Different CLU can bind to different sugar chains.

The main components of TAP detection reagent are condensates (lectin combination), which can agglutinin dozens of TAP to generate crystal-like condensates with specific forms. The image analyzer of TAP detection can be significantly observed, and it is very different from the form formed by normal blood. In this way, we can determine whether or not the subject has TAP in their blood and how much TAP is in their blood.

TAP has great characteristics and advantages as a marker detection. Glycoprotein is mainly distributed on the cell surface, cell endocrine granules, and extracellular matrix. O-sugar chains and *n*-sugar chains, as small molecular substances, can be specifically identified by lectins (lectins combination) and bound by noncovalent bonds, resulting in condensation and precipitation. TAP test can realize the combination detection of more than 20 kinds of abnormal sugar chains related to tumor at one time to gather a variety of tumor signals.

### 2.4. Clinical Significance of TAP Test Results

#### 2.4.1. The TAP Is Positive

The TAP content in the samples was abnormal, and the crystal-like condensate was larger. There are more than 10 cancer cells in the body, and the tumor may not have formed at this time, but the probability of tumor occurrence is significantly higher than that of the tap-negative population. At this point, the patient should be further confirmed with the combination of the medical history, symptoms, signs, other TM tests, and imaging results. Interference factors of TAP positive were excluded. If not, it is recommended to review every two weeks. If the results of three consecutive tests all contain crystal-like condensates, great attention should be paid to them and close observation should be followed up (it is recommended to review every six months). Concerns about chronic conditions can be addressed by using appropriate methods to improve immunity until the TAP test condensates disappear. TAP positive is not necessarily a tumor but can be seen as a warning signal of a high-risk group, which should be paid attention to. Positive people should actively find out the cause, to see whether there is a bad life habits, psychological pressure, and to apply effective health intervention, correction is possible to reverse, such as multiple strong positive should be in-depth clinical examination, in order to find early, early treatment.

#### 2.4.2. Weak Positive TAP

The TAP content in the samples was abnormal, and the crystal-like condensate was small. Body cancer cell number is in 10 10 between and should prevent to turn positive. Eliminate whether there is positive interference disease, pay attention to chronic disease, and improve immunity appropriately.

#### 2.4.3. The TAP Is Negative

The contents of TAP in the samples were normal without obvious agglomerates. This indicates that the number of cancer cells in the body is less than 1 million, which is normal, and the probability of tumor formation within one year is very low. Therefore, TAP test once a year can achieve the purpose of early prevention.

#### 2.4.4. Significance of TAP Expression Changes during and after Treatment

The negative expression of TAP after surgery or other treatment indicates that the tumor may have been completely removed. After TAP negative expression or TAP weak positive expression, if TAP positive expression occurs again within a short period of time, it means that there is a residual tumor or the tumor has metastasized. After a long period of time after the negative expression of TAP, the positive expression of TAP was reestablished, indicating recurrence or metastasis.

## 3. Experimental Methods

### 3.1. Clinical Data

A total of 95 patients diagnosed with thyroid cancer admitted to a hospital from May 2016 to May 2018 were selected as the study objects as the observation group. All the patients had complete clinical and follow-up data, including 60 male patients and 35 female patients, aged 45-75 years. In addition, 55 healthy patients who came to the hospital for physical examination from May 2016 to May 2018 were randomly selected as the control group, including 40 males and 15 females, aged from 30 to 70 years.

Inclusion criteria: the pathological types of patients were confirmed by histopathology. Local lesions cannot be removed surgically, or patients refuse surgery. All patients did not receive any antitumor therapy before enrollment. Cargill score ≥70 can enter the liquid diet at least. Lesion length is <10 cm. The results of routine blood tests in the laboratory were all within the normal range, the electrocardiogram showed no abnormality, and the liver and kidney functions showed no abnormality. No other antitumor therapy was performed recently after radiotherapy, as shown in Table 1.

### 3.2. TAP Detection Method

In this study, tumor laboratory personnel were responsible for TAP test, TAP test comprehensive diagnostic instrument, and TAP test kit at different time points (before treatment and at the end of treatment). The operation was conducted in strict accordance with the operating instructions. Blood samples were taken from the tip of the study object's finger and made into 3 evenly thin blood slices, which were dried naturally. TAP detection reagent was shaken well, and three drops of each sample were added vertically to the blood slices with a dropper. The samples were placed under the TAP integrated slide reader microscope, and the 4 times flat field achromatic objective was used to scan and observe the 3 spots of the blood sample in the display screen at the last time, looking for the agglomerates with specific morphology. The TAP result is judged according to the area of condensate. TAP is in the blood and can be in condensing agent reaction generates specific image; negative image snowflake; dendritic, tree round-shaped, or loose sand; dark brown granules; no visible particle condensed matter, the following as shown in Figure 1(a); and positive condensed particle diameter greater than 38*μ*m^2^, oval, round, or irregular polygon at the edge of the relatively complete crystal sample condensate, as shown in Figure 1.

TAP test reference range: normal TAP/no obvious condensate 0-121 *μ*m^2^; smaller TAP anomaly/condensate, 121-225 *μ*m^2^; and TAP anomaly/condensate was larger, >225 *μ*m^2^.

In addition, 10 mL of patients' fasting peripheral venous blood was collected in the morning and centrifugated at 3000 r/min for 12 min. CEA and SCC levels were detected by automatic electrochemical luminescence immunoassay.

SPSS software package was used to process the statistical data. Measurement data were expressed as mean ± standard deviation, *T*-test was used, and counting data were expressed as percentage. Chi-square test was used, and *P* < 0.05 was considered statistically significant. Correlation analysis of TAP positive expression and short-term efficacy was conducted by Spearman level correlation analysis; *P* < 0.05 was considered statistically significant.

## 4. Discussion

### 4.1. Analysis of TAP Expression in the Two Groups before Treatment

Before treatment, the TAP positive expression rate in the observation group was 74.73% (71/95), significantly higher than that in the control group (10.91% (6/55), with a statistical difference (*P* < 0.05) as shown in Table 2.

### 4.2. Changes of Tumor Markers before and after Treatment

The mean levels of TAP, CEA, and SCC in 95 patients before radiotherapy were 149.33 *μ*m^2^, 2.36 ng/mL, and 1.20 ng/mL, respectively. After radiotherapy, the TAP level was 65.32 *μ*m^2^, significantly lower than that before radiotherapy, and the difference was statistically significant (*P* < 0.01), while CEA and SCC were 2.40 ng/mL and 1.19 ng/mL, respectively, showing no statistically significant difference compared with that before radiotherapy (*P* > 0.05), as shown in Table 3:

### 4.3. Changes of Tumor Markers in Patients with Different Short-Term Effects before and after Treatment

After radiotherapy, the short-term efficacy of 95 patients with thyroid cancer was evaluated as CR in 19 cases (20%), PR in 53 cases (55.7%), and NR in 23 cases (24.2%). The TAP index in PR and CR patients was significantly lower after radiotherapy than before radiotherapy, and the difference was statistically significant (*P* < 0.05). CEA and SCC levels of thyroid cancer patients with the same efficacy evaluation showed no significant difference (*P* > .05) as shown in Table 4 and Figure 2.

### 4.4. Relationship between Different Short-Term Efficacy and TAP

At the end of treatment, esophageal cancer patients with different short-term efficacy showed a difference in TAP after treatment, and the highest in nonremission (NR), followed by partial remission (PR), and the lowest in complete response (CR). However, there was no difference in SCC and CEA results among esophageal cancer patients with different short-term efficacy, as shown in Table 5 and Figure 3.

### 4.5. Analysis of the Correlation between TAP Positive Expression and the Short-Term Efficacy of Treatment

Of the 95 patients in the study, none had serious complications caused by radiotherapy, and all enrolled patients successfully completed the treatment. The short-term efficacy evaluation was mainly based on the results of CT examination. The specific situation of the efficacy evaluation is as follows: complete response (CR) in 19 cases, accounting for 20%. There were 53 cases with partial remission (PR), accounting for 55.7%. There were 23 cases without remission (NR), accounting for 24.2%. Among the 95 patients, statistical analysis showed that there was a statistically significant difference in the effective rate of radiotherapy between those with positive TAP expression and those with negative TAP expression. Statistical Spearman level correlation analysis showed that there was a negative correlation between TAP positive expression and short-term efficacy.

## 5. Conclusions

1. Thyroid carcinoma is a relatively common endocrine gland malignant tumor; if treatment is not appropriate, there will be a high risk of recurrence or metastasis, and abnormal sugar chain glycoprotein (TAP) has a close relationship with the development of the disease; therefore, the purpose of this article is to discuss abnormal sugar chain glycoprotein (TAP) as thyroid cancer curative effect evaluation and radiation and chemotherapy after surgery clinical significance
2. In this study, 95 patients diagnosed with thyroid cancer in a hospital were selected as the study objects and set as the observation group. The clinical and follow-up data of the patients were retrospectively analyzed. Meanwhile, 55 healthy patients were randomly selected as the control group. TAP, squamous cell carcinoma antigen (SCC) level, and carcinoembryonic antigen (CEA) level were detected in peripheral blood of 95 patients with thyroid cancer before and after treatment. The short-term efficacy was evaluated by chest CT examination, and the changes of the three markers before and after treatment and the correlation with the short-term efficacy of the patients were compared
3. The results of this study showed that the level of TAP positive expression in thyroid cancer patients was significantly higher than that in healthy people, suggesting that TAP can be used as a specific indicator for early thyroid cancer screening. After radiotherapy, the TAP positive expression level of patients with thyroid cancer gradually decreased, suggesting that TAP can be used as a specific indicator to determine the short-term efficacy of radiotherapy for thyroid cancer. The short-term radiotherapy effect of thyroid cancer patients is negatively correlated with the positive expression level of TAP protein. Thyroid cancer patients with high TAP protein have poor short-term radiotherapy effect, suggesting that this factor can be used as an indicator to predict the short-term radiotherapy effect of thyroid cancer patients. The detection of TAP positive expression in thyroid cancer patients before radiotherapy can better predict the short-term efficacy and has high clinical value. Clinicians can make individualized treatment plans according to the different expressions of this factor in different patients

## Figures and Tables

**Figure 1:** TAP detection image.

**Figure 2:** The changes of tumor markers before and after radiotherapy in patients with thyroid cancer with company's short-term efficacy.

**Figure 3:** The rank sum test of tumor markers before and after radiotherapy for thyroid cancer with the company.

**Table 1:** Distribution of clinical baseline data of 95 patients with thyroid cancer.

Gender	Number of cases	Constituent
Male	60	63.15%
Getting out	35	36.84%

**Table 2:** Expression of TAP in the observation group was compared with that in the control group before treatment.

Group	Number of cases	The TAP	
		Positive	Feminine
Observation group	95	71	24
Matched group	55	6	49
Chi-square value		63.1	
*P* value		<0.001	

**Table 3:** The Changes of tumor markers in patients with thyroid cancer before and after radiotherapy.

	The TAP (*μ*m^2^)	The CEA (ng/mL)	SCC (ng/mL)
Prior treatment	149.33	2.36	1.20
After treatment	65.32	2.40	1.19

**Table 4:** Changes of tumor markers before and after radiotherapy in patients with thyroid cancer with company's short-term efficacy.

Group	Period	The TAP (*μ*m^2^)	The CEA (ng/mL)	SCC (ng/mL)
PR (*n* = 53)	Prior treatment	159.97	2.36	1.30
	After treatment	53.31	2.35	1.27
CR (*n* = 19)	Prior treatment	155.76	2.39	1.17
	After treatment	47.57	2.31	1.13
NR (*n* = 23)	Prior treatment	119.51	2.35	1.01
	After treatment	107.67	2.61	1.35

**Table 5:** Rank sum test of tumor markers before and after radiotherapy for thyroid cancer with company's short-term effects.

The test period and the items		NR	PR	CR
The prior treatment TAP	Mean rank	39.97	49.35	47.36
	*P* value	0.473		
After treatment the TAP	Mean rank	65.11	41.76	39.11
	*P* value	0.002		
The prior treatment CEA	Mean rank	46.35	46.76	51.96
	*P* value	0.793		
After treatment the CEA	Mean rank	51.63	45.19	46.31
	*P* value	0.693		
The prior treatment SCC	Mean rank	37.11	50.03	47.97
	*P* value	0.137		
After treatment SCC	Mean rank	47.65	43.16	48.63
	*P* value	0.793		

## Data Availability

The data in the article are all real and available.
